# Associations between polymorphisms of the *PDLIM4* gene and susceptibility to osteoporotic fracture in an elderly population of Han Chinese

**DOI:** 10.1042/BSR20181505

**Published:** 2019-01-18

**Authors:** Jihang Chen, Zheping Hong, Chen Zhao, Qing Bi, Binsong Qiu

**Affiliations:** 1 Department of Orthopedics, Zhejiang Provincial People’s Hospital, People’s Hospital of Hangzhou Medical College, Zhejiang, PR China; 2 Department of Orthopedics, the Second Affiliated Hospital of Wenzhou, Medical University, Zhejiang, PR China

**Keywords:** bone mineral density, osteoporosis, PDZ and LIM domain protein 4, single nucleotide polymorphism

## Abstract

The aim of the present study was to investigate the associations between single nucleotide polymorphisms (SNPs) in the PDZ and LIM domain protein 4 (*PDLIM4*) gene and susceptibility to osteoporotic fracture in an elderly Han Chinese population. Seven SNPs of *PDLIM4*, including rs77584624, rs78418541, rs270611, rs3900945, rs77486529, rs71583465, and rs366512, were examined in 540 elderly Chinese patients with osteoporotic fractures (case group) and 540 healthy Chinese subjects (control group) using Sanger sequencing. A-allele carriers of rs270611 in PDLIM4 had a significantly high risk of osteoporotic fracture (adjusted odds ratio [OR] = 1.34; 95% confidence interval [CI]: 1.24–1.46; *P*<0.001). Similarly, individuals carrying the C-allele at PDLIM4 rs3900945 were predisposed to osteoporotic fracture (adjusted OR = 1.45; 95% CI: 1.05–1.25; *P*<0.001). In contrast, the T-allele at rs366512 appeared to be a protective genetic factor against osteoporotic fracture (adjusted OR = 0.84; 95% CI: 0.74–0.95; *P*<0.01). Consistently, the serum levels of N-terminal propeptide of type I procollagen (PINP) and C-telopeptide fragments of Collagen type I α1 chains (β-CTx) were higher in A-allele carriers of rs270611 and C-allele carriers of rs3900945, while T-allele carriers of rs366512 had lower PINP and β-CTx levels. Corresponding well with published findings, the A-allele of rs270611 and C-allele of rs3900945 were associated with reduced bone marrow density (BMD) at the fracture site, while T-allele carriers of rs366512 were shown to have normal BMD. Our study provides supportive evidence for the contribution of *PDLIM4* gene polymorphisms to the susceptibility to osteoporotic fracture and suggests that rs270611 and rs3900945 are genetic risk factors, while rs366512 might be a genetic protective factor against osteoporotic fracture in elderly Han individuals.

## Introduction

Osteoporosis is the commonest metabolic bone disease characterized by low bone mass and microarchitectural deterioration of bone tissue, which leads to enhanced bone fragility and greater risk of bone fractures [1]. With rapid economic improvements in society, longer human life expectancy, and lower birth rates, the Chinese population has aged considerably over the past few decades, causing a concomitant increase in the prevalence of ageing-related chronic diseases such as osteoporosis [2–4]. Osteoporosis is associated with increased fracture risk. Hip fracture is the most devastating osteoporotic-related fracture due to the consequent disability, mortality and costs, both personal and societal, causing a substantial public health burden [5].

The pathogenesis and pathophysiology of osteoporosis have not been fully elucidated yet, despite epidemiological studies having indicated that numerous factors might contribute to the etiology of osteoporosis, including a low intake of calcium, vitamin D deficiency, tabacco use, alcohol intake, and lack of exercise etc. [6]. However, these conventional risk factors do not fully account for all the cases. Evidence from genetic studies has suggested that genetic factors are important determinants of bone mass and play crucial roles in the etiology of osteoporosis. Over the past few decades, a number of genes have been found to be associated with susceptibility to osteoporosis, including low-density lipoprotein receptors 5 (LRP5), vitamin D receptor, estrogen receptor, carrier protein E, and type I collagen [7–10]. These factors, separately or in combination, may contribute to increased bone resorption and decreased bone formation.

PDZ and LIM domain protein 4 (*PDLIM4*), localized within the cytokine cluster of chromosome 5 (5q31.1), encodes a protein with the PDZ and LIM domain-containing adapter found in association with the actin cytoskeleton [11,12]. Studies of mouse models and human patients have established that PDLIM4 plays crucial roles in many fundamental biological processes such as cytoskeleton organization, neuronal signaling, cell-lineage specification, and organ development; moreover, pathological processes like oncogenesis and reduced PDLIM4 activity are attributable to many human diseases [13]. PDLIM4 has been reported to be involved in the formation and development of osteoblasts. Single nucleotide polymorphisms (SNPs) are common form of genetic variation within the genome. In a genetic study of 370 adult Japanese women, a significant association was identified between the PDLIM4 genetic variation and radial bone mineral density [14]. We hypothesize that genetic polymorphisms in *PDLIM4* gene might affect bone remodeling capacity and alter the risk of osteoporotic fracture in a specified population. To obtain a comprehensive estimate of the putative influence of the genetic polymorphisms of *PDLIM4* on osteoporotic fracture risk and to obtain genetic evidence for the prevention of the disease, several polymorphisms in *PDLIM4* with minor allele frequencies above 0.05 were detected in this case-control study in a sample population of elderly Han Chinese individuals.

## Materials and methods

### Patient characteristics

This hospital-based case-control study was conducted from May 2015 until December 2017. A total of 540 consecutive patients (285 men, 255 women; 71.6 ± 10.9 years) with a primary diagnosis of osteoporotic fracture were recruited from the Department of Orthopedics, Zhejiang Provincial People’s Hospital. Simultaneously, 540 normal healthy controls (291 men, 249 women; 72.1 ± 9.8 years) were enrolled. All enrolled patients fulfilled the following inclusion criteria: (i) osteoporotic fractures, defined as fractures resulting from fall injuries and having *T*-scores ≤−2.5 at either the femoral neck or spine; (ii) patients who had undergone surgery or conservative treatment; and (iii) patients aged 50 years or above. The exclusion criteria included the following: (i) patients who had severe liver, kidney, or other systemic diseases; (ii) patients who had other metabolic disorders that can affect bone metabolism, including diabetes mellitus, hyperthyroidism, hypothyroidism, and diseases of the pituitary gland; (iii) patients who had undergone surgeries involving the hip or lumbar spine; (iv) patients who had experienced a high-impact injury, such as a traffic accident; and (v) patients with any serious complications, such as lung infections and gastrointestinal bleeding. Written informed consent was obtained from all subjects. The present study was approved by the Ethics Committee of Zhejiang Provincial People’s Hospital (no. 2015031402P).

### Measurement of bone resorption and formation markers

C-telopeptide fragments of Collagen type I α1 chains (β*-*CTx) and N-terminal propeptide of type I procollagen (PINP) are recommended as markers of bone resorption and bone formation, respectively. Serum levels of β-CTx and PINP were determined by an electrochemiluminescence immunoassay (ECLIA) on a Beckman Coulter UniCel DxI 800 system (Beckman Coulter, Germany).

### Bone marrow density measurement

Areal bone marrow density (BMD) (g/cm^2^) was measured by dual-energy X-ray absorptiometry (Hologic^®^, Waltham, MA, U.S.A.) at the L2–L4 vertebrae, femoral neck, and total hip. Results obtained on a Hologic, Inc. 1000 (Hologic Europe, Zaventum, Belgium) or a Norland Medical Systems (Norland Corp., Vaerlose, Denmark) bone densitometer. Results obtained on the Norland Medical Systems densitometer were corrected for the difference between the two densitometers using the correction formulas suggested by Genant et al. [15]. All BMD values were corrected for age and gender.

### DNA extraction and SNP sequencing

Blood samples were obtained from all subjects in the morning while they were in a fasting state. Genomic DNA was isolated with the QIAamp DNA Mini Kit (Qiagen, Hilden, Germany) according to the manufacturers’ instructions. The extracted DNA was diluted in nuclease-free water and stored at −80°C for further use. The *PDLIM4* gene loci rs77584624, rs78418541, rs270611, rs3900945, rs77486529, rs71583465, and rs366512 were examined by Sanger sequencing assay. A 25 μl of PCR reaction system was used, containing 2.5 μl of 10X Taq polymerase buffer solution, 2 μl of magnesium chloride (2 mM), 2 μl dNTP mix (0.2 mM), 1 μl forward primer (10 pmol), 1 μl reverse primer (10 pmol), 2 μl genomic DNA (100 ng/μl), 0.5 μl DNA Taq polymerase enzyme, and 14 μl distilled water. PCR amplification conditions were programmed on a thermocycler (Gene Cycler, Bio-Rad, U.S.A.) as follows: denaturation at 94°C for 4 min; 35 cycles of 94°C for 30 s and 60°C for 40 s; and a final extension cycle at 72°C for 10 min. The primers used for PCR amplification are listed in Table 1. The PCR products were subjected to Sanger sequencing using the Genetic Analyzer Freeware and subsequently analyzed by Minor Variant Finder software (Applied Biosystems, U.S.A.).

**Table 1:** PDLIM4 SNP loci and PCR amplification primers

SNP	MAF*	Primer sequence (5′ -> 3′)
rs77584624	G: 0.1068	Forward primer: GGGATACATTGGGTGGAAGC
		Reverse primer: AACAGTGCAGACCTTTTCTGG
rs78418541	T: 0.1068	Forward primer: CCCTCAGGACAGCCAGTGATA
		Reverse primer: TCCCCAGGACTTAGACCCTA
rs270611	A: 0.2039	Forward primer: GACAATGCAGTGACCAGCTCT
		Reverse primer: GGTTTCTGCTCAGCCCCTTG
rs3900945	C: 0.3495	Forward primer: TTTCTGTGTCCACTCCCACG
		Reverse primer: CCTATGAACCAGGGGCTTGC
rs366512	T: 0.1942	Forward primer: CCCCTCCCCACAAGATGACAC
		Reverse primer: CCTGGGAAACTTGAGGAACGG
rs77486529	G: 0.1068	Forward primer: AGGCCCGTTCCTCAAGTTTC
		Reverse primer: TCCTCAGACTAGCCACGCTC
rs71583465	C: 0.3495	Forward primer: CGGCTGGGCTTTAAGAGACT
		Reverse primer: ATGATTCCACGCTCCACCTG

*: 1000 genomes data from Han Chinese in Beijing. Abbreviation: MAF, minor allele frequency.

### Statistical analysis

Statistical analyses were performed by SPSS 22.0 (SPSS Inc., Chicago, IL, U.S.A.). Qualitative characteristics are presented as numbers and percentages. Numerical data are expressed as mean ± standard error of the mean or standard deviation (SD), or percentages. The hereditary equilibrium was assessed by the Hardy–Weinberg test, and the genotype and allele frequencies of the *PDLIM4* SNPs were evaluated by the chi-square test. Demographic variables between patients and controls were compared by the chi-square test and Student’s *t*-test. The genotype relative risk was calculated using the odds ratio (OR) and a 95% confidence interval (CI). The coefficient (D′) of pairwise linkage disequilibrium (LD) – the non-random association between the SNPs – was calculated using Haploview version 4.2. All *P* values were two sided, and statistical significance was considered at *P*<0.05.

## Results

### Population characteristics

Patient demographics are shown in Table 2. The case group consisted of 540 patients with a primary diagnosis of osteoporotic fracture, amongst which 17.6% of the lesions (95 cases) occurred in the lumbar spine, 30.6% (165 cases) in the thighbone, 22.8% (123 cases) in the proximal humerus, 21.3% (115 cases) in the distal radius, and 7.8% (42 cases) in the thoracic vertebra. The control group included 540 normal healthy controls matched for reproductive age and sex. The baseline characteristics of the two groups indicated that there were no statistically significant differences in age, sex composition, body mass index (BMI), smoking, or alcohol consumption (Table 2).

**Table 2:** Comparisons of baseline characteristics between the case and control group

	Case group (*n*=540)	Control group (*n*=540)	*P* value
Age (years, mean ± SD)	71.6 ± 10.9	72.1 ± 9.8	0.428
Sex [n (%)]			
Male	285 (52.8%)	291 (53.9%)	0.714
Female	255 (47.2%)	249 (46.1%)	
BMI (kg/m^2^, mean ± SD)	22.4 ± 1.8	22.6 ± 1.8	0.068
Smoking status			
Yes	241 (44.6%)	250 (46.3%)	0.582
No	299 (55.4%)	290 (53.7%)	
Alcohol drinking			
Yes	245 (45.4%)	254 (47.0%)	0.583
No	295 (54.6%)	286 (53.0%)	
Fracture site			
Lumbar	95 (17.6%)		
Thighbone	165 (30.6%)		
Proximal humerus	123 (22.8%)		
Distal radius	115 (21.3%)		
Thoracic vertebra	42 (7.8%)		

### Associations between *PDLIM4* gene SNPs and osteoporotic fracture

All genotypic frequencies of our studied SNPs were ascertained in a balanced state in the Han Chinese population, based on the Hardy–Weinberg equilibrium (*P*>0.05). Table 3 summarizes the genotype and allele frequency distributions of *PDLIM4* SNPs (rs77584624, rs78418541, rs270611, rs3900945, rs77486529, rs71583465, and rs366512) between the case and control group. No significant difference was detected in the frequencies of alleles and genotypes of rs77584624, rs78418541, rs77486529, and rs71583465 polymorphisms between the case and control group (*P*>0.05). However, the frequency of the AA genotype of the rs270611 SNP was significantly higher in patients with osteoporotic fracture than in the control subjects (χ^2^ = 58.09; *P*<0.001), and the AA genotype was associated with a significantly increased risk of osteoporotic-related fracture in the dominant (adjusted OR = 1.25; 95% CI: 1.11–1.41; *P*<0.001) and recessive model (adjusted OR = 1.80; 95% CI: 1.60–1.96; *P*<0.001). Individuals carrying the A-allele of the rs270611 SNP were susceptible to osteoporotic fracture (adjusted OR = 1.34; 95% CI: 1.24–1.46; *P*<0.001). A significantly higher frequency of the CC genotype at rs3900945 was found in the case group (χ^2^ = 21.61; *P*<0.001), and this genotype was linked with the susceptibility of osteoporotic fracture in the recessive model (adjusted OR = 1.39; 95% CI: 1.22–1.57; *P*<0.001) but not in the dominant model (adjusted OR = 1.05; 95% CI: 0.93–1.19; *P*=0.50). C-carriers of the rs3900945 SNP were predisposed to osteoporotic fracture (adjusted OR = 1.45; 95% CI: 1.05–1.25; *P*<0.001). There was no significant difference in the genotypic frequencies of the rs366512 SNP between the case and control group (*P*>0.05), whereas the TT genotype was associated with a significantly decreased risk of osteoporotic fracture in the dominant (adjusted OR = 0.85; 95% CI: 0.74–0.97; *P*=0.02) and recessive model (adjusted OR = 1.52, 95% CI: 0.27–0.88; *P*=0.01). The T-allele of the rs366512 SNP was a protective factor for osteoporotic fracture (adjusted OR = 0.84; 95% CI: 0.74–0.95; *P*<0.01).

**Table 3:** Distribution of PDLIM4 polymorphisms and osteoporotic fractures risk

SNP	Case (*n*=540)	Control (*n*=540)	*P* value	Crude OR (95% CI)	*P* value	Adjusted OR (95% CI)
rs77584624						
TT	415 (76.9%)	424 (78.5%)	1.00 (reference)			
TG	119 (22.0%)	107 (19.8%)	0.39	1.14 (0.84–1.54)	0.44	1.07 (0.91–1.22)
GG	6 (1.1%)	9 (1.7%)	0.47	0.68 (0.21–2.11)	0.64	0.81 (0.35–1.37)
TG + GG	125 (23.1%)	116 (21.5%)	0.51	1.10 (0.82–1.48)	0.56	1.05 (0.90–1.20)
TT + TG	534 (98.9%)	531 (98.3%)	1.00 (reference)			
GG	6 (1.1%)	9 (1.7%)	0.44	0.66 (0.21–2.05)	0.60	0.80 (0.35–1.35)
T	949 (87.9%)	955 (88.4%)	1.00 (reference)			
G	131 (12.1%)	125 (11.6%)	0.69	1.06 (0.81–1.38)	0.74	1.03 (0.89–1.16)
rs78418541						
CC	403 (74.6%)	420 (77.8%)	1.00 (reference)			
CT	114 (21.1%)	109 (20.2%)	0.57	1.09 (0.80–1.48)	0.62	1.04 (0.89–1.21)
TT	23 (4.3%)	11 (2.0%)	0.03	2.18 (1.00–4.83)	0.05	1.38 (1.00–1.69)
CT + TT	137 (25.4%)	120 (22.2%)	0.22	1.19 (0.89–1.59)	0.25	1.09 (0.94–1.24)
CC + CT	517 (95.7%)	529 (98.0%)	1.00 (reference)			
TT	23 (4.3%)	11 (2.0%)	0.04	2.14 (0.99–4.73)	0.06	1.37 (0.99–1.67)
C	920 (85.2%)	949 (87.9%)	1.00 (reference)			
T	160 (14.8%)	131 (12.1%)	0.07	1.26 (0.98–1.63)	0.08	1.12 (0.99–1.25)
rs270611						
CC	265 (49.1%)	325 (60.2%)	1.00 (reference)			
CA	175 (32.4%)	194 (35.9%)	0.45	1.11 (0.85–1.45)	0.49	1.06 (0.91–1.22)
AA	100 (18.5%)	21 (3.9%)	<0.001	5.84 (3.47–9.92)	<0.001	1.84 (1.62–2.03)
CA + AA	275 (50.9%)	215 (39.8%)	<0.001	1.57 (1.22–2.01)	<0.001	1.25 (1.11–1.41)
CC + CA	440 (81.5%)	519 (96.1%)	1.00 (reference)			
AA	100 (18.5%)	21 (3.9%)	<0.001	5.62 (3.37–9.43)	<0.001	1.80 (1.60–1.96)
C	705 (65.3%)	844 (78.1%)	1.00 (reference)			
A	375 (34.7%)	236 (21.9%)	<0.001	1.90 (1.56–2.31)	<0.001	1.34 (1.24–1.46)
rs3900945						
TT	235 (43.5%)	247 (45.7%)	1.00 (reference)			
TC	177 (32.8%)	224 (41.5%)	0.17	0.83 (0.63–1.09)	0.19	0.91 (0.78–1.05)
CC	128 (23.7%)	69 (12.8%)	<0.001	1.95 (1.36–2.79)	<0.001	1.33 (1.15–1.52)
TC + CC	305 (56.5%)	293 (54.3%)	0.46	1.09 (0.85–1.40)	0.50	1.05 (0.93–1.19)
TT + TC	412 (76.3%)	471 (87.2%)	1.00 (reference)			
CC	128 (23.7%)	69 (12.8%)	<0.001	2.12 (1.52–2.96)	<0.001	1.39 (1.22–1.57)
T	647 (59.9%)	718 (66.5%)	1.00 (reference)			
C	433 (40.1%)	362 (33.5%)	<0.01	1.33 (1.11–1.59)	<0.01	1.45 (1.05–1.25)
rs366512						
CC	368 (68.%)	329 (60.9%)	1.00 (reference)			
CT	163 (30.2%)	186 (34.4%)	<0.01	0.32 (0.14–0.74)	0.01	0.50 (0.26–085)
TT	9 (1.7%)	25 (4.6%)	0.06	0.78 (0.60–1.02)	0.07	0.89 (0.77–1.01)
CT + TT	172 (31.9%)	211 (39.1%)	0.01	0.73 (0.56–0.94)	0.02	0.85 (0.74–0.97)
CC + CT	531 (98.3%)	515 (95.4%)	1.00 (reference)			
TT	9 (1.7%)	25 (4.6%)	<0.01	0.35 (0.15–0.79)	0.01	0.52 (0.27–0.88)
C	899 (83.2%)	844 (78.1%)	1.00 (reference)			
T	181 (16.8%)	236 (21.9%)	<0.01	0.72 (0.58–0.90)	<0.01	0.84 (0.74–0.95)
rs77486529						
AA	421(78.0%)	431(79.8%)	1.00 (reference)			
AG	108 (20.0%)	101 (18.7%)	0.56	1.10 (0.80–1.50)	0.61	1.05 (0.89–1.21)
GG	11 (2.0%)	8 (1.5%)	0.47	1.41 (0.52–3.87)	0.62	1.17 (0.68–1.61)
AG + GG	119 (22.0%)	109 (20.2%)	0.46	1.12 (0.83–1.51)	0.50	1.06 (0.91–1.22)
AA + AG	529 (98.0%)	532 (98.5%)	1.00 (reference)			
GG	11 (2.0%)	8 (1.5%)	0.79	1.38 (0.51–3.79)	0.64	1.16 (0.68–1.59)
A	950 (88.0%)	963 (89.2%)	1.00 (reference)			
G	130 (12.0%)	117 (10.8%)	0.38	1.13 (0.86–1.48)	0.42	1.06 (0.92–1.20)
rs71583465						
GG	224 (41.5%)	238 (44.1%)	1.00 (reference)			
GC	234 (43.3%)	228 (42.2%)	0.51	1.09 (0.83–1.42)	0.55	1.05 (0.91–1.20)
CC	82 (15.2%)	74 (13.7%)	0.38	1.18 (0.81–1.72)	0.43	1.08 (0.89–1.29)
GC + CC	316 (58.5%)	302 (55.9%)	0.39	1.11 (0.87–1.43)	0.42	1.06 (0.93–1.20)
GG + GC	458 (84.8%)	466 (86.3%)	1.00 (reference)			
CC	82 (15.2%)	74 (13.7%)	0.59	1.13 (0.79–1.61)	0.55	1.06 (0.89–1.24)
G	682 (63.1%)	704 (65.2%)	1.00 (reference)			
C	398 (36.9%)	376 (34.8%)	0.32	1.09 (0.19–1.31)	0.35	1.05 (0.96–1.14)

### Stratification analysis by gender and age for *PDLIM4* gene polymorphisms and osteoporotic fracture risk

We further investigated the associations between the *PDLIM4* gene polymorphisms and osteoporotic fracture risk in a study stratified by gender and age. The results were shown in Tables 4 and 5. When stratified by gender, T-allele carriers of rs366512 was associated with a decreased risk of osteoporotic fracture in females (adjusted OR = 0.82; 95% CI: 0.67–0.99; *P*=0.04) but not in males (adjusted OR = 0.88; 95% CI: 0.72–1.06; *P*=0.18). With regards to other studied loci, this stratified analysis did not obtain positive findings.

**Table 4:** Stratification analysis by gender for PDLIM4 polymorphisms and osteoporotic fractures risk

SNP	Case (*n*=540)	Control (*n*=540)	*P* value	Adjusted OR (95% CI)
rs77584624				
Male				
TT	219 (40.56%)	229 (42.41%)		1.00 (reference)
TG/GG	66 (12.22%)	62 (11.48%)	0.66	1.055 (0.85–1.28)
Female				
TT	196 (36.30%)	195 (36.11%)		1.00 (reference)
TG/GG	59 (10.93%)	54 (10.00%)	0.78	1.042 (0.83–1.27)
rs78418541				
Male				
CC	200 (37.04%)	216 (40.00%)		1.00 (reference)
CT/TT	85 (15.74%)	75 (13.89%)	0.32	1.105 (0.91–1.32)
Female				
CC	203 (37.59%)	204 (37.78%)		1.00 (reference)
CT/TT	52 (9.63%)	45 (8.33%)	0.58	1.075 (0.85–1.32)
rs270611				
Male				
CC	129 (23.89%)	169 (31.30%)		1.00 (reference)
CA/AA	156 (28.89%)	122 (22.59%)	0.00	1.296 (1.09–1.54)
Female				
CC	136 (25.19%)	157 (29.07%)		1.00 (reference)
CA/AA	119 (22.04%)	92 (17.04%)	0.03	1.22 (1.01–1.45)
rs3900945				
Male				
TT	123 (22.78%)	133 (24.63%)		1.00 (reference)
TC/CC	162 (30.00%)	158 (29.26%)	0.60	1.054 (0.89–1.26)
Female				
TT	112 (20.74%)	114 (21.11%)		1.00 (reference)
TC/CC	143 (26.48%)	135 (25.00%)	0.74	1.038 (0.87–1.25)
rs366512				
Male				
CC	199 (36.85%)	187 (34.63%)		1.00 (reference)
CT/TT	86 (15.93%)	104 (12.96%)	0.18	0.878 (0.72–1.06)
Female				
CC	169 (31.30%)	142 (26.30%)		1.00 (reference)
CT/TT	86 (15.93%)	107 (19.81%)	0.04	0.820 (0.67–0.99)
rs77486529				
Male				
AA	218 (40.37%)	231 (42.78%)		1.00 (reference)
AG/GG	67 (12.41%)	60 (11.11%)	0.46	1.087 (0.88–1.31)
Female				
AA	203 (37.59%)	200 (37.04%)		1.00 (reference)
AG/GG	52 (9.63%)	49 (9.07%)	0.93	1.022 (0.80–1.26)
rs71583465				
Male				
GG	112 (20.74%)	121 (22.41%)		1.00 (reference)
GC/CC	173 (32.04%)	170 (31.48%)	0.64	1.049 (0.88–1.26)
Female				
GG	112 (20.74%)	117 (21.67%)		1.00 (reference)
GC/CC	143 (26.48%)	132 (24.44%)	0.55	1.063 (0.89–1.28)

**Table 5.** Stratification analysis by ages for PDLIM4 polymorphisms and osteoporotic fractures risk

SNP	Case (*n*=540)	Control (*n*=540)	*P* value	Adjusted OR (95% CI)
rs77584624				
<60 years				
TT	77 (14.26%)	39 (7.22%)		1.00 (reference)
TG/GG	23 (4.26%)	18 (3.33%)	0.32	0.85 (0.59–1.13)
≥60 years				
TT	338 (62.59%)	385 (71.30%)		1.00 (reference)
TG/GG	102 (18.89%)	98 (18.15%)	0.33	1.09 (0.92–1.27)
rs78418541				
<60 years				
CC	79 (14.63%)	43 (7.96%)		1.00 (reference)
CT/TT	21 (3.89%)	14 (2.59%)	0.75	0.93 (0.64–1.23)
≥60 years				
CC	324 (60.00%)	377 (69.81%)		1.00 (reference)
CT/TT	116 (21.48%)	106 (19.63%)	0.14	1.131 (0.96–1.31)
rs270611				
<60 years				
CC	50 (9.26%)	22 (4.07%)		1.00 (reference)
CA/AA	50 (9.26%)	35 (6.48%)	0.23	0.847 (0.67–1.10)
≥60 years				
CC	215 (39.81%)	304 (56.30%)		1.00 (reference)
CA/AA	225 (41.67%)	179 (33.15%)	<0.001	1.34 (1.17–1.54)
rs3900945				
<60 years				
TT	50 (9.26%)	28 (5.19%)		1.00 (reference)
TC/CC	50 (9.26%)	29 (5.37%)	0.92	0.987 (0.77–1.27)
≥60 years				
TT	185 (34.26%)	219 (40.56%)		1.00 (reference)
TC/CC	255 (47.22%)	264 (48.89%)	0.35	1.07 (0.93–1.24)
rs366512				
<60 years				
CC	55 (10.19%)	25 (4.63%)		1.00 (reference)
CT/TT	45 (8.33%)	32 (5.93%)	0.24	0.85 (0.66–1.10)
≥60 years				
CC	313 (57.96%)	304 (56.30%)		1.00 (reference)
CT/TT	127 (23.52%)	179 (33.15%)	0.01	0.818 (0.70–0.96)
rs77486529				
<60 years				
AA	78 (14.44%)	38 (7.04%)		1.00 (reference)
AG/GG	22 (4.07%)	19 (3.52%)	0.17	0.80 (0.55–1.08)
≥60 years				
AA	343 (63.52%)	393 (72.78%)		1.00 (reference)
AG/GG	97 (17.96%)	90 (16.67%)	0.23	1.11 (0.94–1.30)
rs71583465				
<60 years				
GG	43 (7.96%)	26 (4.81%)		1.00 (reference)
GC/CC	57 (10.56%)	31 (5.74%)	0.88	1.039 (0.81–1.35)
≥60 years				
GG	181 (33.52%)	212 (39.26%)		1.00 (reference)
GC/CC	259 (47.96%)	271 (50.19%)	0.44	1.06 (0.92–1.23)

The stratified analysis by age showed that the A-allele of rs270611 was associated with susceptibility to osteoporotic fracture in the age <60 years group (adjusted OR = 1.34; 95% CI: 1.17–1.54; *P*<0.001) but not in the age ≥60 years group (adjusted OR = 0.85; 95% CI: 0.67–1.10; *P*=0.23). Besides, in group age ≥60 years group, A-allele carriers of rs366512 were correlated a higher risk of osteoporotic fracture (adjusted OR = 1.34; 95% CI: 1.17–1.54; *P*<0.001), whereas T-allele appeared to be a protective genetic factor against osteoporotic fracture in age <60 years subgroup (adjusted OR = 0.82; 95% CI: 0.70–0.96; *P*=0.01).

### Haplotype analysis

As the SNPs rs270611, rs3900945, and rs366512 in *PDLIM4* were significantly associated with osteoporotic fracture risk, we performed a haplotype-based association study specifically based on these three SNPs. The *PDLIM4* SNPs rs270611, rs3900945, and rs366512 were determined to be in linkage disequilibrium (Table 6 and Figure 1). Four main haplotypes were present, including CCC, CTC, ATC, and ATT. Overall, CCC and CTC haplotypes were associated with a higher osteoporotic fracture risk (OR = 3.96; 95% CI : 2.99–5.25; *P*<0.001; OR = 2.74; 95% CI: 2.05–3.66; *P*<0.001), whereas the ATC and ATT haplotypes appeared to show a protective impact against osteoporotic fracture (OR = 0.30; 95% CI: 0.20–0.44; *P*<0.001; OR = 0.56; 95% CI: 0.33–0.94; *P*=0.02).

**Table 6.** Haplotypic association of PDLIM4 gene in Chinese Han elderly patients with osteoporotic-related fracture

Haplotype no.	Haplotype*	Case group	Control group	OR (95% CI)	*P* value
1	CCC	0.489	0.194	3.96 (2.99–5.25)	<0.001
2	CTC	0.378	0.181	2.74 (2.05–3.66)	<0.001
3	ATC	0.081	0.230	0.30 (0.20–0.44)	<0.001
4	ATT	0.048	0.083	0.56 (0.33–0.94)	0.02

*rs270611, rs3900945, rs366512.

**Figure 1:** Linkage disequilibrium tests for *PDLIM4* SNPs (rs270611, rs3900945, and rs366512) in the case group

### Associations between *PDLIM4* gene SNPs and serum β-CTx and PINP levels

We also detected serum β-CTx and PINP levels. Significantly, higher levels of serum β-CTx and PINP were observed in patients with osteoporotic fracture than in control individuals (*P*<0.05). We further studied whether the *PDLIM4* gene SNPs can affect the expression of β-CTx and PINP. The results revealed that the alleles and genotypic distribution of *PDLIM4* showed no significant differences between patients with osteoporotic-related fracture and control subjects. However, data revealed that the AA genotype at rs270611 and the CC genotype at rs3900945 were associated with significantly higher levels of β*-*CTx and PINP, whereas the TT genotype at rs366512 appeared to have reduced serum β-CTx and PINP expression (*P*<0.05) (Figure 2). There was no relationship between the levels of β-CTx and PINP and the genetic variants rs77584624, rs78418541, rs77486529, and rs71583465 in both groups (*P*>0.5).

**Figure 2:** The measurements of serum PINP and β-CTx levels (**A**) Serum PINP levels of the case and control group. (**B**) Plasma levels of serum PINP with the allelic distribution of *PDLIM4* gene variants. (**C**) Serum β-CTx levels of the case and control groups. (**D**) Plasma levels of serum β-CTx with the allelic distribution of *PDLIM4* gene variants.

### Associations between *PDLIM4* gene SNPs and BMD

BMD was also measured in the present study. Patients with osteoporotic fracture exhibited significantly higher total BMD, as well as BMD of L2–L4 vertebrae, femoral neck, and total hip compared with control subjects (*P*<0.05, Figure 3A). No significant association was detected for the *PDLIM4* rs77584624 and rs78418541 SNPs with BMD levels (*P*>0.05, Figures 3B,C). However, individuals carrying the AA genotype at rs270611 and CC genotype at rs3900945 had significantly lower BMD levels (*P*<0.05, Figures 3D,E). Also, there was no association identified between SNPs of rs77486529, rs71583465 and BMD levels (*P*>0.05, Figures 3F,G), whereas the TT genotype at rs366512 appeared to have higher BMD (*P*<0.05, Figure 3H).

**Figure 3:** BMD measurements (**A**) BMD of the case and control groups; (**B–H**) BMD with the allelic distribution of *PDLIM4* gene variants including rs77584624, rs78418541, rs270611, rs3900945, rs77486529, rs71583465, and rs366512.

## Discussion

To our knowledge, this is the first study to estimate the association of *PDLIM4* polymorphisms with osteoporosis susceptibility and prognosis. In the present study, we found that the rs270611 SNP AA genotype and rs3900945 SNP CC genotype were associated with an increased risk of osteoporotic fracture, while the rs366512 SNP played a protective role against osteoporotic fracture development. Data also revealed that the AA genotype at rs270611 and the CC genotype at rs3900945 were associated with significantly higher levels of β-CTx and PINP, whereas the TT genotype at rs366512 appeared to have reduced serum β-CTx and PINP expression.

PDLIM4 was initially identified from the rat fibroblast cells as a tumor suppressor gene that can encodes PDZ and LIM domain proteins [16]. Recent work on the PDZ-LIM protein family has revealed that it has important activities at the cellular level, mediating signals between the nucleus and the cytoskeleton, with significant impact on organ development. Bone morphogenetic protein 6 (BMP-6) is a phylogenetically conserved protein that plays an important role in bone regeneration. LMP-1 is an essential positive regulator of the osteoblast differentiation program as well as an important intermediate step in the BMP-6 signaling pathway [17]. Similarly, PDLIM4 might have participated in osteoblast differentiation and the regulation of bone formation. The molecular mechanism by which the genetic variation induces the alteration in function remains to be fully elucidated.

Thus far, limited research has addressed the association of genetic polymorphisms in *PDLIM4* gene with human diseases. A previous study of Japanese women has shown that the PDLIM4 (-3333T–>C) genetic variation of the 5′-flanking region is associated with radial BMD, suggesting that it may disrupt the function of PDLIM4 and contribute to osteoporosis [14]. To date, the role of *PDLIM4* SNPs in the development of osteoporotic fracture has not been demonstrated. There are multiple SNP loci within *PDLIM4*. According to the data in the 1000 Genomes Project (https://www.ncbi.nlm.nih.gov/variation/tools/1000genomes/), we selected seven SNP loci at *PDLIM4* and examined the genotype frequencies in this case-control study. There was no significant difference in the frequencies of the alleles and genotypes of rs77584624, rs78418541, rs77486529, or rs71583465 polymorphisms between the case and control group, suggesting that these loci might not participate in the development of osteoporotic fracture. Bone turnover markers used to evaluate bone metabolic activity are proposed as alternative indicators for bone mineral density in the diagnosis and management of osteoporosis [18]. Bone metabolism mainly includes the process of bone formation and resorption. Currently, the measurements of serum levels of β-CTx and PINP are recommended as markers of bone resorption and bone formation markers, respectively, correlated with the corresponding histomorphometric parameters of bone formation and resorption [19]. Our results showed that individuals carrying different variants within rs77584624, rs78418541, rs77486529, and rs71583465 have similar serum levels of PINP and β-CTX, as well as BMD, suggesting that the above loci would not affect bone remodeling activity. SNPs of rs77584624, rs78418541, rs77486529, and rs71583465 are located in the non-coding regions of the *PDLIM4* gene, which also have no significant influence on transcription and transmission; therefore, mutations within these loci did not affect bone metabolism or osteoporotic-related fracture.

In the present study, we found that the rs270611 SNP AA genotype and rs3900945 SNP CC genotype were associated with an increased risk of osteoporotic-related fracture, while the rs366512 SNP played a protective role against osteoporotic fracture development. Data also revealed that the AA genotype at rs270611 and the CC genotype at rs3900945 were associated with significantly higher levels of β-CTx and PINP and lower BMD, whereas the TT genotype at rs366512 appeared to have reduced serum β-CTx and PINP expression and higher BMD. It is acknowledged that the SNPs of rs270611 and rs3900945 were located in the encoding regions that would affect PDLIM4 expression, which might participate in the regulation of osteoblast differentiation and bone formation. This corresponds with the finding that the mutant type of rs270611 and rs3900945 SNPs had higher PINP and β-CTx, indicating that individuals carrying the mutant genotypes have active bone turnover processes with the enhancement of bone formation and resorption [20]. Besides, we found that the T-allele of the rs366512 SNP was a protective factor against osteoporotic fracture. The TT genotype at rs366512 appeared to have reduced serum β-CTx and PINP expression and increased BMD. Similarly, the SNP at rs366512 was located in the coding regions of *PDLIM4*. Mutant T-allele carriers appeared to have increased PDLIM4 expression as evidenced by the increased PINP and β-CTx serum levels and low BMD. The exact mechanism by which the variation at the rs366512 locus alters PDLIM4 function is still unclear.

In the stratified analysis, we found that T-allele carriers of rs366512 were associated with a decreased risk of osteoporotic fracture in females but not in males. As osteoporotic fractures were common in postmenopausal women due to estrogen deficiency, the genetic protective factor was believed to play a more important role in the high-risk group. Besides, A-allele of rs270611 was associated with susceptibility to osteoporotic fracture in the age <60 years group but not in the age ≥60 years group. In the age ≥60 years group, A-allele carriers of rs366512 were correlated a higher risk of osteoporotic fracture, whereas T-allele appeared to be a protective genetic factor against osteoporotic fracture in age <60 years subgroup. It might be associated with the imbalance between calcium and phosphorus due to physiological decline of renal function in aged population. Besides, thyroid hormones were key regulators of bone homeostasis in adulthood. Abnormal secretion of thyroid hormones was often observed in old age population, which might oppose a favorable effect on osteoporotic fracture. Together, this finding suggested that the interaction between SNP of rs366512, rs270611, and age was associated with osteoporotic fractures.

Over the past few decades, research on the regulation of PDLIM4 expression has mainly focused on DNA methylation. A significant down-regulation of PDLIM4 expression has been well described in prostate cancer, and the hypermethylation of the *PDLIM4* gene is considered to be associated with the down-regulation. Furthermore, the hypermethylation of *PDLIM4* could be used as a sensitive molecular tool in the detection of prostate tumorigenesis [21]. The hypermethylation of the *PDLIM4* gene was suggested to correlate with the expression of estrogen receptor and progesterone receptor [22]. Furthermore, the functionality of an SNP associated with epigenetic modification has been demonstrated. Promoter SNPs of human potassium chloride co-transporter 3 (SLC12A6) not only affect promoter activity but also motivate the promoter gene to produce an additional DNA methylation site [23]. In the present study, SNPs within rs270611, rs3900945, and rs366512 were found to be linked with the development of osteoporotic fracture. Whether there was a functional link between PDLIM4 genetic variation and PDLIM4 methylation remains to be fully validated in future studies.

Four main haplotypes were present, including CCC, CTC, ATC, and ATT. Overall, CCC and CTC haplotypes were associated with a higher osteoporotic fracture risk, whereas ATC and ATT haplotypes appeared to show a protective impact on osteoporotic fracture. *PDLIM4* is localized on chromosome 5q31.1, a region where genetic variations and linkage interactions widely exist. The high degree of polymorphism of the *PDLIM4* gene has made it valuable for linkage studies to further explore the possible contributions of *PDLIM4* gene polymorphisms to osteoporotic fracture.

## Conclusion

Our study provides supportive evidence for the contributions of *PDLIM4* gene polymorphisms to the susceptibility to osteoporotic fracture and suggests that rs270611 and rs3900945 are genetic risk factors, while rs366512 might be a genetic protective factor against osteoporotic fracture in elderly Han Chinese individuals. Validation by a larger study with more patients and diverse ethnicities is needed to confirm these findings.

## Abbreviations

β-CTx: C-telopeptide fragments of collagen type I α1 chain
BMD: bone marrow density
BMI: body mass index
BMP-6: bone morphogenetic protein 6
CI: confidence interval
LRP5: low-density lipoprotein receptor 5
OD: odds ratio
PDLIM4: PDZ and LIM domain protein 4
PINP: N-terminal propeptide of type I procollagen
SD: standard deviation
SNP: single nucleotide polymorphism
